The article "The Effects of Switching from Sevoflurane to Short-Term Desflurane prior to the End of General Anesthesia on Patient Emergence and Recovery: A Randomized Controlled Trial" was published in 2022. Journal: Biomed Res Int.

# The Effects of Switching from Sevoflurane to Short-Term Desflurane prior to the End of General Anesthesia on Patient Emergence and Recovery: A Randomized Controlled Trial

**DOI:** 10.1155/2022/1812728

**Published:** 2022-07-06

**Authors:** Ji Wook Kim, Jeong Yup Lee, Si Won Hwang, Dong-Hee Kang, Sie Jeong Ryu, Doo Sik Kim, Ju Deok Kim

**Affiliations:** Department of Anesthesiology and Pain Medicine, Kosin University Gospel Hospital, Busan, Republic of Korea

## Abstract

While sevoflurane and desflurane have been regarded as inhalation agents providing rapid induction and emergence, previous studies demonstrated the superiority of desflurane-anesthesia compared to sevoflurane-anesthesia in the postoperative recovery in obese and geriatric patients. We investigated whether a short-term switch of sevoflurane to desflurane at the end of sevoflurane-anesthesia enhances patient postoperative recovery profile in non-obese patients. We randomly divide patients undergoing elective surgery (n = 60) into two groups: sevoflurane-anesthesia group (Group-S, *n* = 30) and sevoflurane-desflurane group (Group-SD, *n* = 30). In Group-S, patients received only sevoflurane-anesthesia until the end of surgery (for >2 hours). In Group-SD, sevoflurane was stopped and switched to desflurane-anesthesia before the completion of sevoflurane-anesthesia (for approximately 30 minutes). We assessed the intergroup differences in the times to get eye-opening, extubation, and a bispectral index of 80 (BIS-80). Group-SD showed significantly shorter times to get eye-opening (438 ± 101 vs. 295 ± 45 s; mean difference, 143 s; 95% confidence interval [CI], 101–183; *p* < 0.001), extubation (476 ± 108 vs. 312 ± 42 s; mean difference, 164 s; 95% CI, 116–220; *p* < 0.001), and BIS-80 (378 ± 124 vs. 265 ± 49 minutes; mean difference, 113 s; 95% CI, 58–168 *p* < 0.001) compared to Group-S. There was no between-group difference in postoperative nausea, vomiting, and hypoxia incidences. Our results suggested that the short-term (approximately 30 minutes) switch of sevoflurane to desflurane at the end of sevoflurane-anesthesia can facilitate the speed of postoperative patient recovery.

## 1. Introduction

Safe and fast patient recovery is essential to inhalation anesthesia [1–3]. Since the level of inhalation anesthetics in the brain is the most critical determinant of patient consciousness/unconsciousness, the speed of increase and decay of inhalation anesthetics in the brain can determine the speed of anesthesia induction and postoperative recovery [4].

The blood solubility of each inhalation anesthetic is the most important pharmacologic factor for determining the speed of induction and recovery of various inhalation agents [5–7]. Sevoflurane and desflurane have been widely used and provide relatively rapid induction and emergence due to their low blood solubilities [8, 9].

Meanwhile, the administered inhalation agent can be distributed in the body and accumulated in the adipose tissue [4]. The accumulated agent can interfere with the decay of the brain level after stopping its administration and ultimately delay postoperative recovery, especially in obese patients. Therefore, choosing an inhalation agent with the lowest solubility would be beneficial in enhancing the decay at the brain level and the recovery in these patients.

Previous studies demonstrated that desflurane has a much lower solubility than sevoflurane and desflurane-anesthesia provides a much faster recovery profile than sevoflurane anesthesia in obese and elderly patients [10–13]. Switching sevoflurane-anesthesia to desflurane-anesthesia after endotracheal intubation also enhanced emergence and postoperative recovery in non-obese patients [14]. However, despite many studies demonstrating the impact of the long-term switch of inhalation agents, it is difficult to find previous studies investigating that of a short-term switch at the end of anesthesia.

We hypothesized that switching sevoflurane to desflurane at the end of sevoflurane anesthesia, even for a brief period, would facilitate postoperative recovery in non-obese patients. Therefore, we randomly compared postoperative recovery profiles in patients who underwent sevoflurane anesthesia and those who switched sevoflurane to desflurane for approximately 30 minutes at the end of sevoflurane anesthesia for thyroid and breast surgery.

## 2. Materials and Methods

### 2.1. Study Design

This single-center, parallel-group, prospective, randomized controlled study was conducted from December 2021 to April 2022. Written informed consent was obtained from all participants; further, this study was approved by the Institutional Clinical Ethics Committee (KUGH-2021-07-49). This trial was registered with the Clinical Research Information Service (KCT0006780) before patient recruitment.

### 2.2. Study Population

We included 60 patients aged 18–65 years with an American Society of Anesthesiologists (ASA) I-II classification who were scheduled to undergo general anesthesia (> 2 h) for elective thyroid and breast surgery. The exclusion criteria were as follows: undergoing total intravenous anesthesia; body mass index ≥30 kg/m^2^; pregnancy or lactation; lung diseases, including asthma and chronic obstructive lung disease; allergy to drugs (including inhalational anesthetics); history of hypersensitivity to remifentanil, other fentanyl analogs, or rocuronium; renal disease (creatinine clearance <60 mL/min or baseline blood creatinine value ≥1.5 mg/dL); liver disease; myasthenia gravis; neuromuscular junction disease; a history of psychiatric disorders, including communication difficulties; a history or family history of malignant hyperthermia; convulsions; and acute hepatic porphyria.

### 2.3. Randomization

This was a randomized trial (random block sizes) with an allocation ratio of 1 : 1. The principal investigator (J.D. Kim) generated a random assignment sequence of the participants using a randomization software (http://www.randomizer.com/) and enrolled the participants. According to the randomization result, the participants were allocated into two groups: sevoflurane-anesthesia group (Group-S); and sevoflurane-desflurane group (Group-SD).

### 2.4. Blinding

The patient, the anesthesiologist responsible for anesthesia administration (researcher A), and the nurse in the anesthesia department were blinded to the group assignment. Another anesthesiologist (researcher B), who was not blinded to the group assignment, received an envelope containing information regarding the group assignment of each patient from the principal investigator, which was used to determine whether only sevoflurane was administered or whether it was switched to desflurane ≥30 minutes before the end of anesthesia. The vaporizer and gas monitor in the anesthesia machine (Dragger Primus, Drager Medical AG & Co KG, Lübeck, Germany) were covered with paper to conceal the anesthetic agent from the researcher B. From the time of switching the inhalational anesthetic to the end of inhalational anesthetic administration, researcher B coordinated the operation of the anesthesia machine including controlling the vaporizer dial according to the bispectral index (BIS) and fresh gas flow rate as instructed by researcher A. All data were assessed by researcher A, and only the minimal alveolar concentration (MAC) value displayed on the anesthesia machine monitor from the time of switching inhaled anesthetic to the end of inhalation anesthetic administration was recorded separately by researcher B.

### 2.5. Anesthesia Regimen

Patients were admitted to the operating room (OR) without pretreatment. Upon entry, basic monitoring equipment (electrocardiography, pulse oximetry, and noninvasive blood pressure) was attached to the patient. The sedation level was evaluated using a BIS sensor (BIS Quatro™ Sensor; Covidien, Mansfield, MA, USA) attached to the patient's forehead. The BIS was measured using a BIS™ Vista A-3000 monitor (Aspect Medical Systems, Inc., Newton, MA, USA). Neuromuscular blockade (NMB) during surgery and recovery was assessed at 15-s intervals using train-of-four (TOF) stimulation of the ulnar nerve with a neuromuscular monitoring device (TOF-Scan®; IDMed; Marseille, France).

Propofol (2 mg/kg) and remifentanil (1 *μ*g/kg) were administered for anesthesia induction. After the loss of consciousness, rocuronium (0.6 mg/kg) was administered to support intraoperative mechanical ventilation. Endotracheal intubation was performed after sufficient muscle relaxation. General anesthesia was maintained through continuous infusion of remifentanil (0.05–0.25 *μ*g/kg/min) and a sevoflurane expiratory concentration of 1.5–2.5%. Additionally, an intraoperative sedation level of BIS 40–60 was maintained. Mechanical ventilation was initiated using an inspired oxygen concentration (FiO_2_, fraction of inspired oxygen) of 50%, a fresh gas flow rate of 4 L/min, a tidal volume of 6 mL/kg, a respiratory rate (RR) of 14 breaths/min, and a positive end-expiratory pressure of 6 cmH_2_O. The RR was appropriately adjusted to maintain an end-tidal carbon dioxide pressure of 35–40 mmHg. The degree of muscle relaxation during surgery was maintained at 2–3 TOF counts. When the TOF count was 4 or more, a bolus of 0.15 mg/kg of rocuronium was administered. For muscle recovery during emergence, rocuronium was not administered for ≥1 hour before the end of surgery.

### 2.6. Interventions

In both groups, sevoflurane was used intraoperatively as an inhalation anesthetic after anesthesia induction. Patients in Group-S received sevoflurane until the end of surgery, while those in Group-SD were switched to desflurane 30 minutes before the end of surgery. The MAC of desflurane was maintained at a constant level shown on the anesthesia monitor immediately before the end of sevoflurane administration.

In both groups, ramosetron (0.5 mg) was intravenously administered 30 minutes before the end of surgery to prevent postoperative nausea and vomiting (PONV). The infusion rate of remifentanil was adjusted to 0.05 *μ*g/kg/min for 10 minutes before the end of the surgery. Administration of inhalational anesthetic agents and remifentanil was stopped at the end of the surgery; additionally, emergence was induced using 100% oxygen with a fresh gas inflow rate of 6 L/min. Subsequently, pyridostigmine was administered to antagonize NMB based on the blockade degree. If the TOF ratio < 0.4, pyridostigmine 200 *μ*g/kg and glycopyrrolate 0.1 mg/kg were administered. If the TOF ratio was ≥0.4, pyridostigmine 100 *μ*g/kg and glycopyrrolate 0.1 mg/kg were administered. In case of the TOF ratio ≥ 0.9, BIS ≥80, and sufficient spontaneous respiration, the endotracheal tube was removed. After monitoring the patient's blood pressure and oxygen saturation for 5 postoperative minutes, the patients were transferred to the PACU.

### 2.7. Data Collection

#### 2.7.1. Primary Outcome Variable

The main evaluation variables were time until eye-opening. The eye-opening time was measured at 10-s intervals from the point when sevoflurane or desflurane was stopped at the end of the surgery until the patient first opened their eyes after verbal instructions from the anesthesiologist. The patient opening their eyes after receiving verbal instructions from the doctor is a method commonly used in clinical practice to assess the patient's recovery after anesthesia. Failure to do so may reflect abnormalities in the brain [15]. In addition, since it has been used as a primary outcome for the evaluation of patient emergence after anesthesia in many studies, it was used in this study as well [8, 14].

#### 2.7.2. Secondary Outcome Variables

The secondary outcome variables included the time to reach a BIS of 80 after discontinuing the anesthetic agent, the BIS value upon eye-opening, the time elapsed from pyridostigmine administration to a TOF ratio of 0.9, and the time to endotracheal extubation. The time to endotracheal tube extubation was defined as the time between stopping sevoflurane or desflurane administration to endotracheal tube removal after sufficient recovery.

MAC with inspiratory/expiratory concentration of inhalation anesthetics, BIS, mean arterial pressure (MAP), and heart rate (HR) were measured at 30-minute intervals for 150 minutes post-induction. Additionally, these values were obtained 10 minutes before and after anesthesia switching, as well as 10 minutes and immediately before the end of anesthesia, to determine the effect of the switching. In Group-SD, the measurements were based on the actual replacement time. In Group-S, it was assumed that the 30 minutes before the end of anesthesia administration corresponded to the replacement time in the Group-SD. The incidence of PONV, dizziness, and hypoxia (O_2_ ≤ 92%) was immediately recorded after extubation and throughout the PACU stay.

### 2.8. Sample Size Calculation

Compared with sevoflurane, desflurane has been found to reduce the time required to recover consciousness after the end of administering inhalation anesthetics by >30% [16]. Our preliminary study showed that the time required to recover consciousness following verbal commands after general anesthesia using sevoflurane was 9.3 ± 3.5 minutes. To evaluate whether replacing sevoflurane with desflurane for 30 minutes before the end of anesthesia would reduce the eye-opening time by >30% (6.6 ± 2.5 minutes with desflurane), we used G-power to identify that 28 participants per group were required to yield *α* = 0.05, power = 0.9, and effect size = 0.89. Considering potential dropouts, we included 60 patients.

### 2.9. Data Analyses

Statistical analyses were performed using PASW Statistics software (version 26.0). The Kolmogorov–Smirnov test was used to examine the distribution normality of continuous data, including the time to eye-opening. We used a two-tailed unpaired Student's *t*-test for between-group comparisons of normally distributed data, with values expressed as the mean and standard deviation. Repeated-measures analysis of variance was used to evaluate between-group differences in the time changes in MAC, BIS, MAP, and HR measured up to 150 min in 30-min intervals. Categorical variables, including the incidence of complications, were examined appropriately using the chi-square test or Fisher's exact test. Statistical significance was set at *p* < 0.05.

## 3. Results and Discussion

### 3.1. Results

Among the 71 eligible patients, five refused to participate; thus, the remaining 66 patients were enrolled and randomly assigned into two groups. Among them, six patients (four in Group-S, two in Group-SD) did not undergo planned intervention since the surgery was completed earlier than the expected 2-h duration. Finally, 30 patients were included in the statistical analysis (see Figure 1). There were no significant between-group differences in the patient baseline characteristics and surgical data (see Table 1).

Compared with Group-S, Group-SD showed a significantly reduced the time to eye-opening and endotracheal tube extubation (see Table 2). There was no between-group difference in the BIS values upon instructed eye-opening; however, Group-SD showed a significantly shorter time to reach a BIS of 80 after inhaled anesthetic discontinuation. There was no between-group difference in the time elapsed from pyridostigmine administration to a TOF ratio of 0.9 (Table 2).

There was no between-group difference in the MAC, inspiratory/expiratory concentration of inhalation anesthetics, BIS, MAP, and HR measured at all aforementioned time points (see Figure 2; Table 3).

There was no between-group difference in post-anesthesia complications or hypoxia as well as the HR and MAP during the PACU stay (Table 4).

## 4. Discussion

Our study showed that compared with Group-S, Group-SD showed a significantly shorter time to eye-opening and extubation, indicating that the short-term switch of sevoflurane to desflurane, at least for 30 min, at the end of sevoflurane anesthesia provides rapid awakening.

Desflurane and sevoflurane are commonly used in our practice. Among all the volatile anesthetics currently used, desflurane has the lowest blood solubility, suggesting the fastest induction and awakening [4]. Despite the advantage of faster recovery, even compared to sevoflurane, undesirable effects, including airway stimulation, tachycardia, and greenhouse effect, can limit the use of desflurane [16–19]. In such cases, sevoflurane can be mostly chosen for anesthesia induction and maintenance due to its little airway stimulation effect. The results of this study can be applied for faster recovery of consciousness in patients who need sevoflurane for anesthesia induction and maintenance. Its application also can be considered for patients requiring immediate postoperative neurological evaluation and prompt patient cooperation after surgery [20].

In the present study, the conversion process was simplified by turning off the sevoflurane vaporizer and turning on the desflurane vaporizer to the target MAC value at the time of switching. In addition, the switching from 0.8 MAC of sevoflurane to desflurane 30 minutes before the end of surgery did not significantly affect the BIS and MAC values from the time of switching till the end of anesthesia. This result provides evidence that can be applied easily in clinical practice. However, changes in the level of sedation due to the switching of the inhalational anesthetics during surgery may differ depending on the type of volatile anesthetic used [21–23]. Therefore, to intraoperatively switch volatile anesthetics, it is necessary to elucidate the characteristics of the volatile anesthetics through the objective determination of their concentration and the level of consciousness.

The result of this study is consistent with that of previous studies on the intraoperative switching use of inhalation anesthetic agents. Mikuni et al. demonstrated that sevoflurane for anesthesia induction and switching to desflurane for anesthesia maintenance within 5 minutes after the induction improves the patients' emergence and recovery profile [14]. Compared with previous study, our study showed that patients could be awakened faster even though the much more extended use of sevoflurane (approximately 5 and 180 minutes, respectively) and relatively shorter use of desflurane (approximately 100 and 30 minutes, respectively). In addition, we measured the level of consciousness during emergence using the BIS value as well as the eye-opening time. The patients who switched to desflurane reached a BIS of 80 and opened their eyes faster than those who received sevoflurane alone; however, there was no between-group difference in the BIS values at the time of eye-opening. In another study, Kang et al. also evaluated the effect of changing isoflurane to desflurane on emergence and recovery in patients undergoing surgery for approximately 3 hours. They reported that replacing isoflurane with desflurane (1 MAC) 1 h before the end of surgery improved emergence and recovery [21]. Based on the results of previous studies and our study, future studies must be conducted on the effects of various long-term surgery on the patient's recovery.

We observed no significant change in the MAP and HR after anesthetic switching, which is also consistent with previous reports [14]. A rapid increase in end-tidal desflurane concentration by >5% was found to induce a transient increase in the HR and blood pressure by inducing sympathetic nerve stimulation [24]. This effect may be noticeable in case of a high fresh gas flow rate and hyperventilation during anesthesia induction [25, 26]. However, in most cases, since sevoflurane was switched with <1 MAC desflurane without high fresh gas flow and hyperventilation, it could be maintained stably without significant changes in the HR and MAP. In addition, even in the PACU, there were no statistical and clinical differences between HR and MAP in patients.

This study has several limitations. First, other than time to eye-opening, we did not clinically evaluate the patients' recovery of consciousness further. Although eye-opening can be one of the important indicators to evaluate the patient's consciousness after surgery and BIS was additionally used in this study, subjective evaluations, including name speaking and handgrip, can allow additional evaluation of recovery of consciousness. Second, the time point for anesthetic switching to desflurane was not the same for all patients since it was difficult to accurately predict the exact surgery duration. Lastly, our study method is applicable when using anesthetic devices equipped with both sevoflurane and desflurane inhalation anesthetic vaporizers.

## 5. Conclusions

In conclusion, in patients under general anesthesia using long-term sevoflurane, switching to desflurane for a 30-minute period before the end of anesthesia can allow rapid recovery of consciousness.

## Figures and Tables

**Figure 1:** Flowchart of patient enrollment.

**Figure 2:** Minimal alveolar concentration (MAC), bispectral index (BIS), mean arterial blood pressure (MAP), and heart rate (HR) values measured in 30-minute intervals up to 150 minutes after induction of anesthesia in both groups. (a) MAC, (b) BIS, (c) MAP, and (d) HR. There was no significant interaction between the two groups over time in MAC, BIS, MAP, and HR by repeated-measures analysis of variance (all *p* > 0.05). Group-S: sevoflurane group; Group-SD: sevoflurane-desflurane group.

**Table 1:** Baseline characteristics and surgical data of the participants.

	Group-S (*n* = 30)	Group-SD (*n* = 30)	*P* value
Sex (M/F)	11/19	12/18	0.791
Age (year)	52.3 ± 10.5	51.9 ± 8.4	0.862
Height (cm)	162.8 ± 8.8	160.4 ± 5.6	0.235
Weight (kg)	61.7 ± 9.3	62.6 ± 9.8	0.731
Body mass index (kg/m^2^)	23.5 ± 2.7	24.4 ± 2.1	0.207
ASA score (I/II)	18/12	16/14	0.602
Duration of surgery (min)	177 ± 59	184 ± 75	0.677
Duration of anesthesia (min)	220 ± 66	227 ± 78	0.683
Fluid infusion (ml)	1508 ± 330	1521 ± 427	0.894
Urine output (ml)	451 ± 280	449 ± 226	0.639
Remifentanil infusion (*μ*g)	810 ± 314	878 ± 477	0.518
Rocuronium dose (mg)	75.4 ± 17.9	75.3 ± 24.9	0.984
*Type of surgery*			
Breast surgery	16	12	
Robotic surgery	5	3	
Non-robotic surgery	11	9	
Thyroid surgery	12	14	
Robotic surgery	2	3	
Non-robotic surgery	10	11	
Others	2	4	

Group-S: sevoflurane group; Group-SD: sevoflurane-desflurane group; ASA: American Society of Anesthesiologists. Data are expressed as mean ± standard deviation or number.

**Table 2:** Emergence variables of the two groups.

	Group-S (*n* = 30)	Group-SD (*n* = 30)	95% CI	*P* value
Time to opening eyes on command (eye-opening) (s)	438 ± 101	295 ± 45	101–183	< 0.001
Time to endotracheal tube extubation (s)	476 ± 108	312 ± 42	116–210	< 0.001
Time to reach BIS 80 (s)	378 ± 124	265 ± 49	58–168	< 0.001
BIS at the time of eye-opening (s)	82.6 ± 4.9	84.6 ± 3.4	-4.4–0.4	0.100
Time from the pyridostigmine to the TOF ratio of 0.9 (s)	340 ± 141	289 ± 83	-28–128	0.204

Eye-opening time: Interval between when the volatile anesthetic was stopped at the end of the surgery and when the patient opened his/her eyes on oral command. Time to endotracheal tube extubation: from stopping administration of the volatile anesthetic and removing the endotracheal tube based on the patient's sufficient recovery. Time to reach BIS 80: the duration from discontinuation of inhalation anesthetic to BIS reach value of 80. BIS at the time of opening eyes: the BIS value when the patient opened their eyes following the doctor's command. Time from pyridostigmine administration to TOF ratio of 0.9: time elapsed from pyridostigmine administration to TOF ratio of 0.9. BIS: bispectral index; TOF: train of four; CI: confidence interval. Data are expressed as mean ± standard deviation.

**Table 3:** Patients' intraoperative data.

	Group-S (*n* = 30)	Group-SD (*n* = 30)	*P* value
Total inhalation anesthetic administration duration (min)	208 ± 66	218 ± 77	0.608
Duration of sevoflurane administration (min)	208 ± 66	180 ± 75	0.227
Duration of desflurane administration (min)	N/A	38 ± 14	
10 minutes before replacement			
MAC (Ins/exp, vol %)	0.81 (1.78/1.55)	0.81 (1.80/1.57)	0.860
BIS	46.4 ± 6.4	43.7 ± 5.3	0.100
MAP (mmHg)	80.5 ± 10.1	78.5 ± 10.6	0.474
HR (beats/min)	66.8 ± 12.4	67.9 ± 12.4	0.749
At the time of replacement			
MAC (Ins/exp, vol %)	0.81 (1.76/1.54)	0.80 (1.79/1.56)	0.765
BIS	45.6 ± 5.6	43.8 ± 6.3	0.243
MAP (mmHg)	79.9 ± 12.3	80.1 ± 10.7	0.962
HR (beats/min)	66.5 ± 12.0	65.5 ± 11.9	0.758
10 minutes after replacement			
MAC (Ins/exp, vol %)	0.81 (1.76/1.54)	0.82 (4.93/4.23)	0.733
BIS	46.3 ± 5.9	43.6 ± 6.2	0.096
MAP (mmHg)	80.9 ± 12.8	78.0 ± 9.9	0.367
HR (beats/min)	66.2 ± 13.0	63.4 ± 10.3	0.371
10 minutes before end of surgery			
MAC (Ins/exp, vol %)	0.79 (1.74/1.53)	0.80 (4.9/4.2)	0.884
BIS	47.6 ± 6.0	44.7 ± 6.6	0.086
MAP (mmHg)	80.6 ± 11.4	76.7 ± 12.4	0.225
HR (beats/min)	64.7 ± 12.7	61.4 ± 8.9	0.277
At the end of surgery			
MAC (Ins/exp, vol %)	0.77 (1.70/1.50)	0.77 (4.80/4.23)	0.914
BIS	49.0 ± 6.3	47.4 ± 7.7	0.376
MAP (mmHg)	81.2 ± 13.7	79.8 ± 10.5	0.681
HR (beats/min)	67.1 ± 12.3	64.8 ± 11.2	0.469

Group-S: sevoflurane group; Group-SD: sevoflurane-desflurane group; MAC: minimal alveolar concentration; Ins/exp vol%: inspiratory and expiratory concentration of sevoflurane and desflurane; BIS: bispectral index; MAP: mean arterial pressure; HR: heart rate; TOF: train of four; N/A: not applicable. Data are expressed as mean ± standard deviation.

**Table 4:** Post-anesthesia care unit data.

	Group-S (*n* = 30)	Group-SD (*n* = 30)	95% CI	*P* value
Fentanyl (*μ*g)	71.4 ± 34.5	64.6 ± 40.3	14.0–27.7	0.512
Desaturation (<92% in pulse oximetry) (*n*)	0	0		
Nausea (*n*)	1	2		0.500
Vomiting (*n*)	0	0		
After 10 min in the PACU				
HR (beats/min)	86.2 ± 15.3	83.2 ± 9.6	− 4.2–10.3	0.407
MAP (mmHg)	96.7 ± 17.2	102.2 ± 12.9	− 14.2–3.1	0.203
After 20 min in the PACU				
HR (beats/min)	82.7 ± 16.9	80.8 ± 10.2	− 6.1–10.0	0.630
MAP (mmHg)	97.9 ± 17.1	100.2 ± 13.1	− 11.0–6.4	0.601

PACU: post-anesthesia care unit; HR: heart rate; MAP: mean arterial pressure. Data are expressed as mean ± standard deviations or number.

## Data Availability

The data that support the findings of this study are available on request from the corresponding author. Due to privacy and ethical concerns, the data cannot be made available to the public.
